# MicroRNA-103a-3p enhances sepsis-induced acute kidney injury via targeting CXCL12

**DOI:** 10.1080/21655979.2022.2062195

**Published:** 2022-05-05

**Authors:** Gaihong Ding, Jinhua an, Luyao Li

**Affiliations:** Department of Nephrology, Xuchang University Medical College, Xuchang City, Henan Province, China

**Keywords:** microRNA-103a-3p, C-X-C motif chemokine 12, sepsis-related kidney injury

## Abstract

Acute kidney injury (AKI) is a common and fatal complication in inflammatory sepsis. Several microRNAs (miRNAs or miRs) have been identified to control sepsis. MiR-103a-3p has been reported to take part in the various inflammatory response. However, its role in AKI remains unclear. The present research aimed to explore the role and mechanisms of miR-103a-3p in AKI. Neurogenic sepsis mouse model and lipopolysaccharide-induced HK-2 and 293 cell models were established. The renal functions in each group of mice were measured. After evaluating the biological functions of C-X-C motif chemokine 12 (CXCL12) and miR-103a-3p on HK-2 and HEK-293 T cells, their interaction was determined. Detection of CXCL12 and apoptosis and inflammation-related factors in renal tissue was done. MiR-103a-3p was significantly repressed in the sepsis model, while CXCL12 was elevated. Furthermore, miR-103a-3p inversely controlled CXCL12. Knockdown of miR-103a-3p or overexpression of CXCL12 could significantly inhibit the progression of HK-2 and HEK293 cells, whereas elevated miR-103a-3p or knockdown of CXCL12 showed the opposite effects. Collectively, miR-103a-3p heightens renal cell damage caused by sepsis by targeting CXCL12.

## Introduction

Sepsis is a systemic inflammatory responding syndrome induced via fungi, bacteria, or viruses, and it results in shock, multi-organ dysfunction syndrome, and death [1]. Acute kidney injury (AKI) is a common and severe complication in sepsis. According to various reports, sepsis facilitates the production of inflammatory cytokines in kidney tissue, thus resulting in kidney cell apoptosis and AKI [2]. Sepsis-induced AKI is associated with the aberrant expression of various genes. Moreover, AKI can be mitigated by effectively regulating the expression of these aberrant genes [3]. Therefore, further research on the pathogenesis of AKI can provide further insight to enhance treatment and improve the survival rates in sepsis-induced AKI patients.

MicroRNAs (miRNAs or miRs) are tiny endogenous RNAs that modulate gene expression after transcription [4,5]. Several human illnesses are linked with miRNA dysregulations. Thus, understanding miRNAs roles may offer new approaches for early diagnosis of diseases and promising targeted therapies [6–8]. For instance, miRNAs play crucial functions in the formation and maintenance of normal kidney physiology. Previous reports indicated that miRNAs play vital functions in AKI’s pathogenesis [9,10]. Therefore, well-designed miRNA-based studies on AKI may drive the development of new diagnostic tools and therapeutic interventions. Microarray analysis showed that the miR-103 expression level was elevated in the plasma of hypertension patients compared to the healthy subjects [11]. Similarly, diabetes mellitus patients’ urine expressed elevated miR-103 than healthy controls [12]. In addition, enhanced circulating miR-103a-3p level was implicated in renal injury in patients with hypertension together with angiotensin II–infused mice [13]. It has also been reported that miR-103a-3p expression was elevated in serum and liver of septic mice, whereas miR-103a-3p inhibition regulated lipopolysaccharide (LPS)-stimulated septic liver damage by suppressing apoptosis, inflammation, and oxidative stress [14]. Nevertheless, the roles and mechanisms of miR-103 in the stimulation of sepsis-induced AKI remain unknown.

C-X-C motif chemokine 12 (CXCL12), a ligand of the G protein-coupled receptor or C-X-C motif chemokine receptor 4 (CXCR4), is implicated in various cellular functions, including tissue cell homeostasis, immune surveillance, and inflammatory reactions [15]. According to Shen *et al*. [16], miR-301a-5p mediates the CXCL12/CXCR4 pathway and regulates acute exacerbations of long-term interceptive pulmonary illness. It has been demonstrated that the expression of CXCL12 and CXCR4 in the kidney increases after ischemia/reperfusion induction of AKI [17].

Endotoxins, which are gram-negative bacterial LPSs, are extensively applied for inducing sepsis models [18]. The research was designed to evaluate miR-103a-3p’s manifestation and its anti-inflammatory and anti-apoptotic effects in a cecal ligated mouse model and LPS-induced cell models. The present study also investigated the miR-103a-3p-related molecular mechanisms in LPS-stimulated human proximal tubular epithelial cells (HK-2). The current results assured miR-103a-3p inhibited inflammation and LPS-stimulated HK-2 cell apoptosis via regulation of the pro-inflammatory gene CXCL12.

## Materials and methods

### Animals and ethical statement

The animal experiment was approved by the Experimental Animal Management Committee of the Experimental Animal Center of Xuchang University Medical College (Approval Number: NC20156033c). In total, 12 clean-grade adult Kunming mice (age, 6–8 week-old; weight, 18–22 g) were purchased from the Experimental Animal Center of Xuchang University Medical College. The animals were randomly divided into two groups, namely the sham (n = 6) and the model (n = 6).

### Cecal ligation and puncture (CLP) model

Sepsis induction was done by CLP as described elsewhere [19]. Before and after the operation, normal saline (0.5 ml)was injected into mice’s tail veins in the sham and model groups. All the mice were exposed to an overnight fasting with free access to water before the experiment. Mice were anesthetized using 0.3% pentobarbital sodium (30 mg/kg) injected intraperitoneally, and the abdomen was disinfected using iodophor. An incision of approximately ~1 cm was made on the abdominal wall along the mid-abdominal line. Ligation of the cecum was done using sterile forceps, while blood vessels of the ileum and cecum were kept away from the middle of the cecum. The cecum was ligated with the sterile target with perforation. The cecum content was extracted, while the appendix and its contents were pushed back into the abdominal cavity. The abdominal wall was eventually sutured. In the sham group, the cecum was not ligated or perforated. Mice were sacrificed 24 h after surgery. All mice were euthanized by CO_2_ asphyxiation (the flow rate of CO_2_ was 30–70% of the chamber volume per minute). Next, the kidney was dissected, removed, and weighed. Half of the kidney tissue was then fixed in formaldehyde solution for the microscopic test. The remaining kidney tissue was stored at −80°C for further experiments.

### Hematoxylin and eosin (H&E) staining

The kidney tissue sections were dewaxed in xylene, embedded in paraffin, and hydrated. The tissue samples were then stained using hematoxylin solution for 5 min and soaked five times in 1% acidic ethanol (1% hydrochloric acid into 70% ethanol). Next, the sections were stained in eosin solution, dehydrated with ethanol, and soaked in xylene. The sections were finally mounted and observed in a light microscope for the pathological morphology of kidney tissues.

### Cell culture and transfection

Human kidney tubular epithelial cells-2 (HK-2) and human embryonic kidney (HEK)-293 cells were purchased from BioVector NTCC (Haidian, Beijing, China). The cells were cultured in DMEM supplemented with 10% fetal bovine serum in 37°C and 5% CO_2._ The cells were grown to a confluence of 70% and passaged for subsequent assays. The cells at a logarithmic growth phase were obtained and divided into two groups. One group was treated with LPS (5 mg/l) to induce inflammation, while only DMEM was added in the second group, followed by incubation. The cells were co-transfected with CXCL12 small interfering (si)-RNA (si-CXCL12), miR-103a-3p inhibitors, miR-103a-3p mimics, or relevant negative controls (NC), using Lipofectamine 2000 (Invitrogen, USA) according to the manufacturer’s guidelines. The cells were then incubated for 24 h in a fresh culture media. Monitoring of the transfection efficiencies was then done through Western blot to determine whether inhibition or up-regulation was successful.

### Reverse transcription-quantitative polymerase chain reaction (RT-qPCR)

Extraction of total RNA was done using the BioZOL reagent (Hangzhou Bioer Technology Co., Ltd, Hangzhou, China), according to the manufacturer’s instructions. The RNA samples’ purity and concentration were determined using the spectrophotometer NanoDrop2000 (Thermo Fisher Scientific, USA). The reverse transcription of the RNA into complementary DNA (cDNA) was done using SYBR Prime Script™ RT-PCR kit (Sigma, St Louis, MO, USA) following the manufacturer’s instruction. Primer 5.0 software was utilized to design the primers, which were synthesized by Takara. The primer-specific sequences are described in Table 1. The RT-qPCR was done using the ExScript™ RT-PCR kit (Takara Holdings, Kyoto, Japan) and the ABI7500 qPCR instrument (Thermo Fisher Scientific, USA). U6 was considered a loading control for miR-103a-3p, with GAPDH for CXCL12. Gene expression data were calculated using the 2^−ΔΔCq^ method.

**Table 1.** Primer design

Name	Primer sequences (5’-3’)
MiR-103a-3p	F: AGCAGCAUUGUACAGGGCUAUGA
	R: AUAGCCCUGUACAAUGCUGCUUU
CXCL12	F: TGCATCAGTGACGGTAAACCA
	R: CACAGTTTGGAGTGTTGAGGAT
U6	F: GCTTCGGCAGCACATATACTAAAAT
	R: CGCTTCACGAATTTGCGTGTCAT
GAPDH	F: TATGATGATATCAAGAGGGTAGT
	R: TGTATCCAAACTCATTGTCATAC

miR, microRNA; CXCL12, C-X-C motif chemokine 12; F, forward, R; reverse.

### Cell Counting Kit-8 (CCK-8) assay

The HK-2 cells in the logarithmic proliferation phase were trypsinized for 2 min at 37°C to a single cell suspension. The cells were re-suspended in 1 mL media and counted. Next, a 100 µl suspension containing 2 × 10^3^ cells was introduced in every well of a 96-well culture plate. The cells were grown for 24, 48, and 72 h. Later, 10 μL CCK-8 from the CCK-8 assay kit (Dojindo, Tokyo, Japan) was added and incubated for 4 h, according to the manufacturer’s instructions. The absorbance was then determined in a microplate reader at an absorption wavelength of 450 nm. Each assay was done in triplicates.

### TUNEL assay

The apoptosis of kidney cells was studied through the TUNEL Assay Kit (KeyGEN BioTECH, Jiangsu, China) according to the manufacturer’s guidelines. The cell samples were deparaffinized, hydrated, and the sections were washed in PBS. Samples were then treated with the proteinase K working solution. After that, sections were incubated with a TUNEL reaction mixture for 60 min at 37°C, followed by culturing with DAPI for 10 min. The samples were observed and analyzed using the fluorescence microscope (Olympus, Japan), and the renal tubular cell apoptosis rate was calculated.

### Western blotting

Extraction of proteins from cells was done through the radio-immunoprecipitation assay (RIPA) lysis buffer and PMSF. Protein concentration determination was based on the bicinchoninic acid protein assay kit (Thermo Fisher Scientific, USA) according to the manufacturer’s instructions. The extracted sample protein was diluted in loading buffer, boiled, and denatured. The proteins were then separated using the 10% SDS-PAGE, and the protein electro-blot was then transferred onto a nitrocellulose membrane and blocked using 5% skim milk. The membrane was later incubated with primary antibodies against Bcl-2 (cat. no. ab32124), Bax (cat. no. ab53154), CXCL12 (cat. no. ab229846) (all 1: 1,000), and GAPDH (cat. no. ab8245; 1: 2,000) (all from Abcam). The membrane was then washed with Tris-buffered saline with Tween 20 buffer and incubated using Horseradish peroxidase-labeled secondary antibody (Abcam, 1:5000). The protein bands were finally detected using chemiluminescence reagent and Bio-rad Gel Dol EZ imager (Gel DOC EZ IMAGER, Bio-rad, California, USA). The developed bands were analyzed using Image J software. The experiment was repeated three times, and the data were averaged.

### ELISA

Mice in sham and CLP groups were sacrificed, the kidney was quickly excised, washed using buffer solution, and homogenized. Tissue homogenate centrifugation was done for 10 min at 12,000 × g. The proteins concentration in kidney homogenate was measured through BCA assay. TNF-α and IL-1β inflammatory cytokines expressions were analyzed using the TNF-α (#KHC3011) and IL-1β (#KAC1211) human enzyme-linked immunosorbent assay (ELISA) kits (Invitrogen Life Biotechnologies, Carlsbad, CA, USA), according to the manufacturer’s instruction, with a microplate reader for measurement of the absorbance at 450 nm. Concentrations of TNF-α and IL-1β were calculated using the standard curves. The results obtained were presented as the amount (pg) of TNF-α and IL-1β per mL of supernatant.

### The luciferase activity assay

The PicTar (pictar.mdc-berlin.de/), miRanda (www.microrna.org), and TargetScan (www.targetscan.org), online bioinformatics tools were used in predicting the binding site of miRNA-103a-3p with CXCL12. Relative luciferase activity was determined through dual-luciferase reporter analysis experiments. Target segments were designed for wild-type (wt) and mutant (mut) CXCL12, and were integrated into the pGL3 plasmid, thus constructing pGL3-CXCL12-wt (CXCL12-wt) and pGL3-CXCL12-mut (CXCL12-mut) reporter plasmids. The HK-2 cells in the logarithmic growth phase were then obtained and plated in a 96-well culture plate. When the cell density was about 70%, the cells were co-transfected with CXCL12-wt, CXCL12-mut, miR-103a-3p mimics, or their NC using the Lipofectamine 2000® transfection reagent (Invitrogen, USA), as per the manufacturer’s guidelines. Next, cells were further incubated for 48 h, and the luciferase activity was investigated via the Dual-Luciferase Reporter Assay System (Promega, Madison, Wisconsin, USA). The experiment was repeated three times, and the average was determined.

### Statistical analysis

Data analysis was done using SPSS19.0 software (IBM Corp.). Data were presented as mean ± standard deviation (SD); a comparison of statistical difference between two groups was made using the Student’s t-test. P < 0.05 was considered statistically significant.

## Results

### MiR-103a-3p is inhibited in mouse kidney tissues in sepsis-induced acute kidney injury

In exploring the role of miR-103a-3p in sepsis-induced kidney injury, a mouse model of sepsis-initiated kidney damage with cecal ligation perforation was established. According to the H&E staining results, the kidney tubules were deformed, interstitial edema was prominent, and renal tubular epithelial cells exhibited apoptosis or necrosis in the model compared to the sham group (Figure 1(a)). The results also revealed that the cecal ligation and puncture group showed significantly increased kidney index than the sham group (P < 0.05; Figure 1(b)). Analysis of the kidney function indicators was also done. The observations indicated significantly increased blood urea nitrogen in the CLP compared to the control group (Figure 1(c)). The serum creatinine was also increased in the CLP than the sham group (P < 0.05; Figure 1(d)). These results indicated that the kidney injury model was successfully established. Furthermore, the analysis of TNF-α and IL-1β was done using the ELISA technique. The results confirmed significant TNF-α and IL-1β elevation in the CLP model compared to the sham group (P < 0.05; Figure 1(e,f)). Further, the expression of miR-103a-3p was analyzed using RT-qPCR. The results indicated significantly down-regulated miR-103a-3p expression in the CLP than in the sham group (P < 0.05; Figure 1(g)). The western blot determination of proteins confirmed significantly higher Bax but lowered Bcl-2 expressions in the kidney tissues of CLP than in the sham mice. (Figure 1(h)). The findings confirm that miR-103a-3p is inhibited in sepsis-induced acute kidney injury in mouse kidney tissues.

**Figure 1.** Detection of renal function-related indicators for mice as well as miR-103a-3p expression in kidney tissue.

### MiR-103a-3p elevates the proliferation of LPS-stimulated HK-2 and HEK-293 T cells

To ascertain the function of miR-103a-3p in sepsis-related kidney damage, HK-2 and HEK293cells were co-transfected with LPS, LPS+ miR-NC, LPS+miR-103a-3p mimic, or LPS+miR-103a-3p inhibitor. The expressions of miR-103a-3p was then determined using RT-qPCR. According to the results, miR-103a-3p expression was significantly reduced in the LPS treated cells compared to controls in both HK-2 and HEK293 cells (Figure 2(a, b)). Cell viability was then analyzed using the CCK-8 assay, and the observations indicated that elevated miR-103a-3p could significantly drive HK-2 and 293 cell proliferation compared to the miR-NC (Figure 2(c,d), p<0.05). The apoptosis analysis through TUNNEL assay showed significantly reduced cell apoptosis in LPS+miR-103a-3p mimic, while miR-103a-3p inhibition significantly elevated apoptosis in both HK-2 and 293 cells (P < 0.05; Figure 2(e-f)). Images of the corresponding HK-2/293 cell cultures are shown in Figure 2(g).

**Figure 2.** MiR-103a-3p elevates the proliferation of LPS-stimulated HK-2 and HEK-293 T cells.

Reverse transcription-quantitative PCR was utilized for detecting the miR-103a-3p expression level after transfection with miR-103a-3p mimics together with inhibitors in LPS-induced; (a) HK-2 and (b) 293 cells. Cell Counting Kit-8 assay was utilized for detecting the function of LPS in (c) HK-2 and (d) 293 cell activities after transfection with miR-103a-3p mimics and inhibitors. TUNEL was utilized for detecting (e) HK-2 and (f) 293 cell apoptosis induced by LPS after transfection with miR-103a-3p mimics and inhibitors. (g) HK-2 and 293 cell culture images. The results are presented as the mean ± standard deviation (n = 3) and were analyzed with Student’s t-test. miR, microRNA; LPS, lipopolysaccharide.

### CXCL12 is a downstream target of miR-103a-3p

In studying the downstream molecular mechanism of miR-103a-3p in AKI, bioinformatics analysis was conducted using the TargetScan database. The data indicated that CXCL12 contains a conserved binding site for miR-103a-3p (Figure 3(a)). RT-qPCR was then used to detect CXCL12 mRNA in the tissues of CLP and sham mice. The observations confirmed significantly increased CLP expression in the CLP mice than in the control group (Figure 3(b)). Moreover, RT-qPCR assay results confirmed significantly increased CXCL12 mRNA expressions in the LPS groups of both HK-2 and HEK293 cells compared to the controls (Figure 3(c, d)). Investigation of the targeted binding of miR-103a-3p and CXCL12 indicated that miR-103a-3p mimics significantly decreased the CXCL12-wt luciferase activity, whereas they had no effects on CXCL12-mut luciferase activity (Figure 3(e)). Furthermore, LPS-dependent augmenting of miR-103a-3p in HK-2 and HEK293 cells significantly decreased CXCL12 expression at the mRNA level compared to the LPS+ miRNA mimics cells (figure 3(f)). Nevertheless, the miR-103a-3p inhibitors significantly increased the CXCL12 mRNA expressions in the HK-2 and HEK293 cells compared to the LPS+ miRNA inhibitors group (Figure 3(g)). Analysis of miR-103a-3p expression confirmed no significant effect on miR-103a-3p after LPS-induced upregulation of CXCL12 or after LPS-induced silencing of CXCL12 in HK-2 and HEK293 cells, compared to the controls (Figure 3(h,i)). Briefly, these observations demonstrate that CXCL12 is a downstream target of miR-103a-3p.

**Figure 3.** CXCL12 is a downstream target of miR-103a-3p.

(a) TargetScan database showed the complementary base pairing for miR-103a-3p and CXCL12. (b) RT-qPCR was used for detecting CXCL12 mRNA levels in CLP mouse tissues. RT-qPCR was utilized to detect CXCL12 mRNA level in (c) HK-2 and (d) 293 cells induced by LPS. (e) Luciferase reporter assay was employed for detecting the binding association between miR-103a-3p and CXCL12. After being transfected with (f) miR-103a-3p mimics or (g) inhibitors, RT-qPCR was utilized for detecting CXCL12 mRNA level on LPS-induced HK-2 and 293 cells. (h and i) After overexpression of CXCL12, RT-qPCR was utilized for detecting the miR-103a-3p level in HK-2 and 293 cells induced by LPS (n = 3). The results are presented as the mean ± standard deviation (n = 3) and were analyzed with Student’s t-test. miR, microRNA; LPS, lipopolysaccharide; RT-qPCR, reverse transcription-quantitative PCR; CXCL12, C-X-C motif chemokine 12.

### Elevated CXCL12 expression inhibits LPS-induced HK-2 and HEK293 cells progression

To further determine the effects of CXCL12 on sepsis-induced kidney injury, HK-2 and HEK293 cells were treated with LPS to establish an *in vitro* kidney injury model. RT-qPCR was then used to determine CXCL12 expression post-sepsis induction. As per the results, CXCL12 expression was significantly increased in the LPS-treated cells than the control groups in HK-2 and HEK293 cells (Figure 4(a,b)). Viability studies results through CCK-8 showed a significant reduction in the population of viable cells in the LPS+CXCL12 compared to the controls in both HK-2 and HEK293 cells. This observation was reversed in the LPS+sh-CXCL12 cells (Figure 4(c,d)). The TUNNEL assay results also confirmed significantly increased apoptosis in the LPS+CXCL12 compared to the LPS+NC or LPS+sh-CXCL12 in both HK-2 and HEK293 cells (Figure 4(d,e)). These results clarified that augmenting of CXCL12 significantly inhibited cell progression.

**Figure 4.** Elevated CXCL12 expression inhibits LPS-induced HK-2 and HEK293 cells progression.

After overexpression and downregulation of CXCL12, reverse transcription-quantitative PCR was utilized for detecting the CXCL12 mRNA level on LPS-induced; (a) HK-2 and (b) 293 cells. (c and d) After overexpression and downregulation of CXCL12, Cell Counting Kit-8 assay was utilized for detecting cell activity. (e and f) After overexpression and downregulation of CXCL12, cell apoptosis was measured via TUNEL (n = 3). The results are presented as the mean ± standard deviation (n = 3) and were analyzed with Student’s t-test. CXCL12, C-X-C motif chemokine 12; LPS, lipopolysaccharide.

### CXCL12 reverses the enhancive effect of miR-103a-3p on LPS-induced HK-2 and 293 cells’ growth

Finally, to clarify the miR-103a-3p-dependent CXCL12 functional regulation in AKI, a CXCL12 overexpression plasmid was transfected in HK-2, and HEK293 cells were transfected with LPS+miR-103a-3p mimics, LPS+miR-103a-3p mimics/CXCL12 or LPS. RT-qPCR was then used to determine miR-103a-3p expression. The results confirmed that miR-103a-3p was significantly increased in LPS+miR-103a-3p mimics and LPS+miR-103a-3p mimics/CXCL12 compared to the LPS group in HK-2 and HEK293 cells (Figure 5(a,b)). The RT-qPCR results for CXCL12 analysis showed significantly increased CXCL12 expression in the LPS+miR-103a-3p mimics/CXCL12 than in the LPS+miR-103a-3p mimics or LPS group in both HK-2 and HEK293 cells (Figure 5(c,d)). The cell viability studies confirmed significantly reduced viable cells in LPS+miR-103a-3p mimics/CXCL12 than in LPS+miR-103a-3p mimics group in both HK-2 and HEK293 cells (Figure 5(e,f)). However, the apoptosis study results confirmed significantly increased apoptosis rate in LPS+miR-103a-3p mimics/CXCL12 compared to LPS+miR-103a-3p mimics group in both HK-2 and HEK293 cells (Figure 5(g,h)). The western blot assessment confirmed increased CXCL12 expression in LPS+miR-103a-3p mimics/CXCL12 than in LPS+miR-103a-3p mimics or LPS group in the kidney tissues of the model mice, which are consistent with the in vitro results (Figure 5(i)). In summary, these observations confirmed that CXCL12 reverses the enhancive effect of miR-103a-3p on LPS-induced HK-2 and 293 cells’ growth.

**Figure 5.** CXCL12 reverses the enhancive effect of miR-103a-3p on LPS-induced HK-2 and 293 cells’ growth.

(a-d) After co-transfecting with miR-103a-3p mimics and CXCL12 overexpression plasmid, reverse transcription-quantitative PCR was utilized to detect miR-103a-3p and CXCL12 mRNA levels in cells. (e and f). After co-transfecting with miR-103a-3p and CXCL12 overexpression plasmid, the Cell Counting Kit-8 assay was utilized for detecting cell activity. (g and h) After co-transfecting with miR-103a-3p and CXCL12 overexpression plasmid, cell apoptosis was detected using a TUNEL assay. (i) Western blotting was used to analyze the CXCL12 protein levels in kidney tissue of model mice. The results are presented as the mean ± standard deviation (n = 3) and were analyzed with Student’s t-test. miR, microRNA; CXCL12, C-X-C motif chemokine 12.

## Discussion

Sepsis is a disease characterized by uncontrolled inflammation due to severe infection. Several studies have found that miRNAs could modulate abnormal inflammatory reactions by reducing inflammatory elements, indicating that miRNAs may have a crucial function in sepsis’ inflammatory reactions and immune modulation. Previous studies confirmed that miRNA expression in sepsis patients’ serum is altered compared to the healthy subjects [20,21]. Vasilescu et al. [22] demonstrated the variation in miRNA expression in the serum of sepsis patients and healthy individuals. The study found that miR-150, miR-182, and miR-486 expressions are significantly changed in sepsis patients. Furthermore, Wang *et al*. [23] revealed that miR-146a and miR-233 expressions were reduced in the serum of sepsis patients.

The present study affirmed that miR-103a-3p was downregulated in CLP-treated mouse models and LPS-stimulated cells, which revealed that miR-103a-3p might be used as a biomarker for detecting and treating sepsis or sepsis-induced AKI. In addition, a recent study suggested miR-103a-3p was downregulated in the blood of pneumonia patients and LPS-stimulated lung cells, while miR-103a-3p overexpression attenuated LPS-stimulated inflammation and enhanced LPS-induced lung epithelium cell activity. Therefore, the present study evaluated LPS-stimulated HK-2 and HEK293 cell viability and apoptosis. It was confirmed that miR-103a-3p reduced cell apoptosis and increased cell viability, thereby indicating that miR-103a-3p elevates sepsis-induced AKI.

The cytokines production leads to cascades of effects in the onset of sepsis, including pro-inflammatory factors such as TNF-α, IL-1β, and IL-6 [24,25]. Reduced TNF-α, IL-1β, IL-8, and IL-6 can boost cell-mediated immune response and enable defense functions to down-regulate infections [26]. TNF-α is characterized by early and quick release to initiate the defense mechanism, whereas changes in TNF-α level could mirror changes in other inflammatory factors [27]. However, IL-6 serves as a cytokine cascade activator, mirroring the association between host inflammatory reaction and disease severity, and acts as a sepsis prognostic marker [28](28). The present study confirmed enhanced TNF-α, IL-1β, and miR-103a-3p expressions in sepsis-induced AKI.

CXCL12 is generally considered a standard pro-inflammatory factor that activates immune cells and attracts them to the inflammatory site through the CXC motif, CXCRs, CXCR4/fusin, and CXCR7 [29]. Previous evidence confirmed that the CXCL12/CXCR4 axis facilitates autocrine-mediated angiogenesis and extends the necessary arteries for kidney vascular formulation [30]. According to previous reports, during early or late diabetic nephropathy, glomerular podocytes can secrete CXCL12, and inhibition of CXCL12 can significantly reduce glomerulosclerosis and proteinuria in patients with type 2 diabetes [31]. Zhao *et al*. [32] reported that high expression of CXCR4/CXCL12 has a role in the pathogenesis of systemic lupus erythematosus. The present study found that CXCL12 is enhanced in LPS-stimulated HK-2 and HEK293 cells. Furthermore, elevated CXCL12 can drive cell apoptosis and reduce cell proliferation activity. This finding is consistent with a previous study on CXCL12 in AKI [33]. In addition, CXCL12 is a target of miR-103a-3p, which can reduce LPS-stimulated inflammation and apoptosis in HK-2 cells by combining with CXCL12. Therefore, miR-103a-3p could protect HK-2 cells from LPS-stimulated damage through the CXCL12/CXCR4 axis.

Meanwhile, reports have confirmed elevated CXCL12 and CXCR4 in the kidneys after ischemia/reperfusion stimulation of AKI. This could be implicated in cell migration to damaged kidney cells. Therefore, the CXCL12/CXCR4 axis is considered the primary target in renal repair. Thus, the miR-103a-3p/CXCL12/CXCR4 axis mechanism provides new insights for the treatment of AKI. In summary, the present results emphasize a distinct miRNA-mediated enhancive mechanism for sepsis: miR-103a-3p alleviates sepsis-related AKI by regulating CXCL12. A detailed mechanism is supposed to help increase survival rates and optimize therapies against AKI in the future.

## References

[1] Wang H, Zhang P, Chen W, et al. Serum microRNA signatures identified by Solexa sequencing predict sepsis patients’ mortality: a prospective observational study. PloS one. 2012;7(6):e38885.2271997510.1371/journal.pone.0038885PMC3376145

[2] Shum H-P, Kong HH-Y, Chan K-C, et al. Septic acute kidney injury in critically ill patients–a single-center study on its incidence, clinical characteristics, and outcome predictors. Ren Fail. 2016;38(5):706–716.2698162110.3109/0886022X.2016.1157749

[3] Tanemoto F, Mimura I. Therapies targeting epigenetic alterations in acute kidney injury-to-chronic kidney disease transition. Pharmaceutic. 2022;15(2):123.10.3390/ph15020123PMC887707035215236

[4] Wang K, Ren Y, Liu Y, et al. miR-4262 promotes proliferation and invasion of human breast cancer cells through directly targeting KLF6 and KLF15. Oncol Res. 2017;25(2):277–283.2762925710.3727/096504016X14732514133203PMC7840800

[5] Zhou S, Xiong M, Dai G, et al. MicroRNA-192-5p suppresses the initiation and progression of osteosarcoma by targeting USP1. Oncol Lett. 2018;15(5):6947–6956.2973186810.3892/ol.2018.8180PMC5920969

[6] Karagkouni D, Paraskevopoulou MD, Chatzopoulos S, et al. DIANA-TarBase v8: a decade-long collection of experimentally supported miRNA–gene interactions. Nucleic Acids Res. 2018 Jan 4;46(D1):D239–D245.2915600610.1093/nar/gkx1141PMC5753203

[7] Rasmussen MH, Lyskjær I, Jersie-Christensen RR, et al. miR-625-3p regulates oxaliplatin resistance by targeting MAP2K6-p38 signalling in human colorectal adenocarcinoma cells. Nat Commun. 2016;7(1):12436.2752678510.1038/ncomms12436PMC4990699

[8] Thomson DW, Dinger ME. Endogenous microRNA sponges: evidence and controversy. Nat Rev Genet. 2016;17(5):272–283.2704048710.1038/nrg.2016.20

[9] Liu Z, Wang S, Q-s M, et al. MicroRNAs in pathogenesis of acute kidney injury. Nephron. 2016;134(3):149–153.2732275810.1159/000446551PMC5089907

[10] Brandenburger T, Lorenzen JM. Diagnostic and therapeutic potential of microRNAs in acute kidney injury. Front Pharmacol. 2020;11:657.3247713210.3389/fphar.2020.00657PMC7240101

[11] Karolina DS, Tavintharan S, Armugam A, et al. Circulating miRNA profiles in patients with metabolic syndrome. J Clin Endocrinol Metab. 2012 Dec;97(12):E2271–6.2303206210.1210/jc.2012-1996

[12] Pordzik J, Jakubik D, Jarosz-Popek J, et al. Significance of circulating microRNAs in diabetes mellitus type 2 and platelet reactivity: bioinformatic analysis and review. Cardiovasc Diabetol. 2019;18(1):1–19.3147085110.1186/s12933-019-0918-xPMC6716825

[13] Lu Q, Ma Z, Ding Y, et al. Circulating miR-103a-3p contributes to angiotensin II-induced renal inflammation and fibrosis via a SNRK/NF-κB/p65 regulatory axis. Nat Commun. 2019;10(1):1–14.3108618410.1038/s41467-019-10116-0PMC6513984

[14] Zhou YP, Xia Q. Inhibition of miR‐103a‐3p suppresses lipopolysaccharide‐induced sepsis and liver injury by regulating FBXW7 expression. Cell Biol Int. 2020;44(9):1798–1810.3236922710.1002/cbin.11372PMC7496651

[15] García-Cuesta EM, Santiago CA, Vallejo-Díaz J, et al. The role of the CXCL12/CXCR4/ACKR3 axis in autoimmune diseases. Front Endocrinol. 2019;27(10):585.10.3389/fendo.2019.00585PMC671845631507535

[16] Shen W, Weng Z, Fan M, et al. Mechanisms by which the MBD2/miR-301a-5p/CXCL12/CXCR4 pathway regulates acute exacerbations of chronic obstructive pulmonary disease. Int J Chron Obstruct Pulmon Dis. 2020;15:2561.3311647310.2147/COPD.S261522PMC7585268

[17] Zuk A, Gershenovich M, Ivanova Y, et al. CXCR4 antagonism as a therapeutic approach to prevent acute kidney injury. Am J Physiol Renal Physiol. 2014;307(7):F783–F797.2508052310.1152/ajprenal.00685.2013

[18] Wang Y, Zhang W, Yu G, et al. Cytoprotective effect of aquaporin 1 against lipopolysaccharide‑induced apoptosis and inflammation of renal epithelial HK‑2 cells. Exp Ther Med. 2018;15(5):4243–4252.2973181910.3892/etm.2018.5992PMC5920784

[19] Sunahara S, Watanabe E, Hatano M, et al. Influence of autophagy on acute kidney injury in a murine cecal ligation and puncture sepsis model. Sci Rep. 2018;8(1):1050.2934841210.1038/s41598-018-19350-wPMC5773584

[20] Fouda E, Midan DAE, Ellaban R, et al., The diagnostic and prognostic role of MiRNA 15b and MiRNA 378a in neonatal sepsis. Biochem Biophys Rep. 2021;26:100988.3381735310.1016/j.bbrep.2021.100988PMC8010206

[21] Szilágyi B, Fejes Z, Pócsi M, et al. Role of sepsis modulated circulating microRNAs. Ejifcc. 2019;30(2):128.31263389PMC6599195

[22] Vasilescu C, Rossi S, Shimizu M, et al. MicroRNA fingerprints identify miR-150 as a plasma prognostic marker in patients with sepsis. PloS one. 2009;4(10):e7405.1982358110.1371/journal.pone.0007405PMC2756627

[23] Wang J-F, Yu M-L, Yu G, et al. Serum miR-146a and miR-223 as potential new biomarkers for sepsis. Biochem Biophys Res Commun. 2010;394(1):184–188.2018807110.1016/j.bbrc.2010.02.145

[24] Moraes CA, Santos G, D’Avila JC, et al. Activated microglia-induced deficits in excitatory synapses through IL-1β: implications for cognitive impairment in sepsis. Molec neurobio. 2015;52(1):653–663.10.1007/s12035-014-8868-525257696

[25] Morita Y, Masters EA, Schwarz EM, et al. Interleukin-27 and its diverse effects on bacterial infections. Front Immunol. 2021;12:1752.10.3389/fimmu.2021.678515PMC816526234079555

[26] Zhao H, Wu L, Yan G, et al. Inflammation and tumor progression: signaling pathways and targeted intervention. Signal Transduct Target Ther. 2021;6(1):1–46.3424814210.1038/s41392-021-00658-5PMC8273155

[27] Schumacher SM, Naga Prasad SV. Tumor necrosis factor-α in heart failure: an updated review. Curr Cardiol Rep. 2018;20(11):1–11.3025919210.1007/s11886-018-1067-7PMC6311126

[28] Liu S, Wang X, She F, et al. Effects of neutrophil-to-lymphocyte ratio combined with interleukin-6 in predicting 28-day mortality in patients with sepsis. Front Immunol. 2021;12:757.10.3389/fimmu.2021.639735PMC800786833796105

[29] Janssens R, Struyf S, Proost P. The unique structural and functional features of CXCL12. Cell Mol Immunol. 2018;15(4):299–311.2908291810.1038/cmi.2017.107PMC6052832

[30] Murad HA, Rafeeq MM, Alqurashi TM. Role and implications of the CXCL12/CXCR4/CXCR7 axis in atherosclerosis: still a debate. Ann Med. 2021;53(1):1598–16123449449510.1080/07853890.2021.1974084PMC8439212

[31] Romoli S, Angelotti ML, Antonelli G, et al. CXCL12 blockade preferentially regenerates lost podocytes in cortical nephrons by targeting an intrinsic podocyte-progenitor feedback mechanism. Kidney Int. 2018;94(6):1111–1126.3038504210.1016/j.kint.2018.08.013PMC6251974

[32] Zhao L-D, Liang D, X-n W, et al. Contribution and underlying mechanisms of CXCR4 overexpression in patients with systemic lupus erythematosus. Cell Mol Immunol. 2017;14(10):842–849.2766594710.1038/cmi.2016.47PMC5649106

[33] Song A, Jiang A, Xiong W, et al. The role of CXCL12 in kidney diseases: a friend or foe? Kidney Dis. 2021;7(3):176–185.10.1159/000514913PMC821601734179113

